# Key Experimental Factors of Machine Learning-Based Identification of Surgery Cancellations

**DOI:** 10.1155/2021/6247652

**Published:** 2021-02-20

**Authors:** Fengyi Zhang, Xinyuan Cui, Renrong Gong, Chuan Zhang, Zhigao Liao

**Affiliations:** ^1^School of Management, Guangxi University of Science and Technology, Liuzhou, Guangxi Province 545006, China; ^2^Business School, Sichuan University, Chengdu, Sichuan Province 610000, China; ^3^School of Economics and Management, Harbin Institute of Technology, University Town, Nanshan, Shenzhen, China; ^4^West China Hospital, Sichuan University, Chengdu, Sichuan Province 610000, China; ^5^West China School of Public Health and West China Fourth Hospital, Sichuan University, Chengdu, Sichuan Province 610000, China

## Abstract

This study aimed to provide effective methods for the identification of surgeries with high cancellation risk based on machine learning models and analyze the key factors that affect the identification performance. The data covered the period from January 1, 2013, to December 31, 2014, at West China Hospital in China, which focus on elective urologic surgeries. All surgeries were scheduled one day in advance, and all cancellations were of institutional resource- and capacity-related types. Feature selection strategies, machine learning models, and sampling methods are the most discussed topic in general machine learning researches and have a direct impact on the performance of machine learning models. Hence, they were considered to systematically generate complete schemes in machine learning-based identification of surgery cancellations. The results proved the feasibility and robustness of identifying surgeries with high cancellation risk, with the considerable maximum of area under the curve (AUC) (0.7199) for random forest model with original sampling using backward selection strategy. In addition, one-side Delong test and sum of square error analysis were conducted to measure the effects of feature selection strategy, machine learning model, and sampling method on the identification of surgeries with high cancellation risk, and the selection of machine learning model was identified as the key factors that affect the identification of surgeries with high cancellation risk. This study offers methodology and insights for identifying the key experimental factors for identifying surgery cancellations, and it is helpful to further research on machine learning-based identification of surgeries with high cancellation risk.

## 1. Introduction

Surgery cancellation is a well-recognized health care quality problem that harms patients and wastes resources, leading to considerable losses for medical institutes and the entire health care system [1–3]. It forces scarce operative resources to remain idle and hinders patients' access to operative services [4]. Estimates of this revenue loss range between USD 1,430 and USD 1,700 for each cancelled case in US hospitals not on a fixed annual budget [5, 6]. In a review of surgery cancellations worldwide [4], the global cancellation rate (CR) generally ranges from 4.65% to 30.3%, which is a high proportion that urgently needs to be reduced. Identification of surgeries with high cancellation risk could provide information for health care service management and enable the adoption of preventive actions for achieving a lower CR [4]. Hence, it is of great value to identify surgeries with high cancellation risk.

For reflecting relevant information on patients and medical operation institutions, the hospital information system (HIS) plays an important role in health care service management, including surgery scheduling. Nowadays, health care service management-related studies on HISs have been conducted in many important fields [7–16], such as research on hospital admission rates [7, 8], clinical medication rules [9, 10], and referral management in hospitals [11, 12]. Particularly, the study of HIS in the field of identification of surgeries with high cancellation risk has proved that applying HIS data to identify surgeries with high and low risks of cancellation is feasible [4].

To date, most surgery cancellation studies have mainly focused on the predictors or risk factors of surgery cancellation. In the risk-factor-based category of cancellation, surgery cancellations generally include institutional resource-, capacity-, and patient-related cancellations. A significant percentage of surgery cancellations could be avoided, according to risk-factor-based analysis [17–19]. The risk factors of surgery cancellation include patient, admission, workup, and surgery schedule information, as well as administrative issues and surgery process records [4, 17, 20–26].

In recent years, various studies have focused on reducing surgery cancellation [21, 27–30]. For example, a team of researchers [27] used discrete event simulation modeling to represent perioperative processes and tested the effects of three scenarios on the number of surgical cancellations. Another team [28] simulated an anesthesiology preoperative assessment clinic to quantify the impact of patient information deficiency to mitigate the problem of surgery delay or cancellation. These studies used industrial engineering techniques to investigate means for reducing the number of surgical cancellations across the system but did not focus on identifying surgery with high cancellation risk. Among the works focusing on identifying surgeries with high cancellation risk, a retrospective cohort study [29] examined the association between patient, surgeon, and system factors and proved that several patient and system factors can be used to identify surgeries with a high likelihood of cancellation. The factors associated with surgery cancellation have been evaluated using chi-squared tests and multivariate logistic regression analyses [21]. Using multilevel logistic regression, an observational cohort study [30] identified patient- and hospital-level factors associated with cancellation owing to inadequate bed capacity. However, the accuracy of the above-mentioned studies only using traditional statistics models is low [29].

Machine learning is a powerful and effective tool for medical study. Machine learning has seen many applications in the fields of health care management [31–33], health care cost prediction [34, 35], and health care insurance [36–38]. Various machine learning models, which are of better performance compared with traditional statistics models, have been used in the field of identification of surgeries with high cancellation risk as well [4]. Particularly, Luo et al. [4] used sampling methods to handle the imbalance of the distribution of cancellation. Considering the performance of feature selection used in health care services [39, 40], Liu et al. [41] developed predictive models of last-minute surgery cancellation, in which forward selection was used as a feature selection method. However, there is no research that measured the effects of feature selection strategy, machine learning model, and sampling methods on the identification of surgery with high cancellation risk and identified the key factors of it.

This study aimed to provide effective methods for the identification of surgeries with high cancellation risk based on machine learning models and analyzed the key factors that affect the identification performance. One-side Delong test and sum of square error analysis were conducted to measure the effects of feature selection strategy, machine learning model, and sampling method on the identification of surgeries with high cancellation risk. This study offers methodology and insights for identifying the key experimental factors for identifying surgery cancellations, and it is useful to further research on machine learning-based identification of surgeries with high cancellation risk, in designing experimental process.

The rest of the paper is organized as follows.  Section 2 provides detailed information about data collection and preparation, the methods used in this study, and model setup. The third part summarizes the experimental results.  Section 4 further discusses the experiment and presents the findings. In Section 5, we draw conclusions from the findings and point out the direction of future work.

## 2. Data and Methods

### 2.1. Data

The data of this study were based on HIS sourced from West China Hospital, which is the largest hospital in southwest China. There are 70 operation rooms in West China Hospital nowadays, most of them usually open from 8 a.m. to 8 p.m., and daily average opening hours reach 12 hours. Overall, the data contained 5,125 cases from January 1, 2013, to December 31, 2014, of which 810 were cancelled (positive) and 4,315 were not, providing a CR of 15.80%. The hospital implemented the surgery day system. In this system, the surgeon has main surgery days; that is, the surgeon has the priority to use the operating room and its equipment on these days. All surgeries were scheduled one day in advance, and after confirmation, medical staff (surgeon, anesthesiologist, and nurse), the operation room, and the patient are bundled together. All cancellations were of institutional resource- and capacity-related types. Apart from the features originally obtained from HIS, we designed some features, according to the experience and knowledge of senior health care managers in West China Hospital, and they are whether the surgeon had surgery before (WSHSB), whether the surgery day was a legal holiday (WSDLH), whether it was the main surgery day (WMSD), whether surgeries have been cancelled (WC), and the number of days admitted (NDA). All the collected features of surgeries are listed in Table 1.

In the following experiment process, we considered not only the relationship between predictors and surgery cancellations but also the accessibility of predictors. As a result, 14 related predictors (features) were preliminarily refined, as described in Table 2, which covered all five information categories mentioned above. Among them, surgery schedule information contained five predictors: operating room (OR), surgeon, number of surgeries in the OR on a day (NSOD), the order number of surgery (ONS), and WSHSB. Then, patients' information and administrative issues contained three predictors each. For patients' information, they were age, sex, and anesthesia type (AT). For administrative issues, they were WSDLH, WMSD, and WC. Subsequently, workup and admission information contained two predictors and one predictor, respectively. Workup information contained WHSB and surgery type (ST), whereas admission information contained NDA.

### 2.2. Methods

The methods used in this study are introduced in the following three aspects: feature selection strategies, machine learning models, and sampling methods.

#### 2.2.1. Machine Learning Models

Considering that the objective of this study is to identify surgery cancellation based on historical HIS data and different predictors, we modeled it as a supervised classification problem and utilized a representative set of machine learning models: random forest (RF), logistic regression (LR), extreme gradient boosting-tree (XGBoost-tree), support vector machine-linear (SVM-linear), and neural networks (NNET).

RF is a classifier composed of an ensemble of decision trees for training and predicting, which is widely used in medical management [42–44]. It is known for the high predictive performance and ability to find complex interactions among features [41, 45]. LR, a classification algorithm derived from linear regression, is a common approach employed in prediction and reasonable benchmark for evaluating other models. Compared with SVM and NNET, it has better interpretability that is important for model understanding and interpretation. XGBoost is an improved algorithm based on the gradient boosting decision tree with more detailed classification, XGB-Linear and XGB-tree. As for XGB-tree, it can construct boosted trees efficiently and when performing node splitting, the gain calculation of different predictors can be performed in parallel. SVM-linear is a kind of generalized linear classifier. Because of its advantages of solving high-dimensional pattern recognition problems and high accuracy, it is applied in this study. NNET is a model like the human brain's ability to predict and categorize, which learns the relationship between independent variables and dependent variables. Nowadays, it has been successfully applied in the classification and prediction of biological and medical data [46–48].

#### 2.2.2. Feature Selection Strategies

This study takes four commonly used feature selection strategies into consideration, and they were forward selection strategy, backward selection strategy, LASSO-based strategy, and importance-based strategy. Forward selection starts with an empty set and iteratively adds the most important feature to the target feature subset from the candidate feature set, while backward selection iteratively removes the least important feature from the candidate feature set [49]. LASSO-based strategy refers to the cost function of the linear regression model added with the constraint of the L1 norm. It uses the control parameter for variable selection and complexity adjustment and is widely used in the medical field [50]. As for the importance-based strategy, RF, an excellent classifier model that has good applicability for feature selection [51, 52], was used to generate a dataset of the importance of each feature after training, and features with positive importance were considered as the most useful features to model training. Hence, feature selection using RF was conducted to select the useful predictors for the identification of the surgeries with high cancellation risk.

#### 2.2.3. Sampling Methods

This study involves three sampling methods: oversampling, undersampling, and original sampling. Oversampling was intended to extract negative samples with replacement until the number of them was consistent with the number of positive samples. Conversely, undersampling extracted positive samples without replacement until their number was the same as the negative samples. Both methods change the class distribution of training data and have been used to address class imbalance [53]. These methods have performed well in several fields, such as in churning predictions related to bank credit cards [54] and classifying poor households [55]. Meanwhile, original sampling is the sampling of the original data set without making changes.

### 2.3. Experiment Setup

Figure 1 shows the entire experimental process mentioned below. For the preliminarily determined 14 related predictors, they may not certainly lead to the best performance of identification of surgery cancellation. Hence, the four feature selection strategies mentioned above (forward selection strategy, backward selection strategy, LASSO-based strategy, and importance-based strategy) were considered to achieve better performance. Subsequently, for a certain strategy, *N* predictors were obtained. To a large extent, the value of *N* is different for each strategy. Hence, predictors selected by original strategy (i.e., no feature selection is conducted) and four different feature selection strategies were applied to the following experiments, respectively.

All samples were divided into two sets, the train and test sets, at a ratio of 8 : 2. Based on this division, the train set was divided into the actual train and the validation sets, at a ratio of 6 : 2. Because of the imbalance in the positive-negative ratio (2 : 11) of the actual train set, we employed not only the original sampling but also over- and undersampling to achieve better performance. The train set and the actual train set were used to train the machine learning models; the validation set was used to determine the hyperparameters of models; and the test set was employed to validate the performance of the machine learning models. For each model, we performed a fivefold cross validation against the test set, nested within which was a fourfold cross validation against the validation set. Cross-validation methods are used to generate folds randomly, which refer to the combination of training and test data subset splits for training and validating machine learning models [56].

In this study, we designed 75 schemes (i.e., 5 × 5 × 3; five feature selection strategies, five machine learning models, and three sampling methods correspond to each other, as mentioned above), and each scheme was run to obtain the performance metrics of the test set. Fivefold cross validation was performed for each scheme to find and validate the optimal model with the best performance. Hence, 375 results of experiments were obtained eventually, from which the scheme with the best performance could be found and the influence of the factors (i.e., feature selection strategy, machine learning model, and sampling method) in surgery cancellation forecasting could be evaluated.

As the identification of surgeries with high cancellation risk in this study belongs to the binary classification problem, the performance of identification was measured according to seven metrics: accuracy, sensitivity, specificity, positive predictive value (PPV), negative predictive value (NPV), net reclassification index (NRI), and area under the curve (AUC) of the receiver operating characteristic (ROC). Sensitivity, specificity, PPV, and NPV are the metrics for model evaluation, which are used to reflect performance in a certain aspect. Sensitivity refers to the ratio of the correctly predicted positive sample number to the total number of true positive samples; conversely, specificity refers to the ratio of correctly predicted negative samples to the total number of true negative samples. Meanwhile, both PPV and NPV are metrics that focus on predictive samples. PPV refers to the ratio of the number of correctly predicted positive samples to the number of predicted positive samples, whereas NPV refers to the ratio of the number of correctly predicted negative samples to the number of predicted negative samples. Accuracy, NRI, and AUC are all used to reflect the overall performance of the model. Accuracy is the ratio of the correctly predicted sample number to the total predicted sample number. It does not distinguish the predicted sample as positive or negative. NRI is a measure of the change in risk prediction obtained when the risk marker under evaluation is added to an existing risk prediction model [57]. It was intended to serve as a summary measure to highlight the difference between two models [58]. AUC considers the imbalance of positive and negative samples and is often used with the ROC curve to illustrate performance assessments so that sensitivity and specificity can be considered in a comprehensive manner. In addition, feasibility is defined as the ability to make a considerable identification, and robustness refers to the measured performance close to the essential performance. In this study, AUC was considered to be the key metric; feasibility and robustness both focus on AUC.

The mentioned metrics were firstly analyzed for top schemes, and then we analyzed statistics (mean, maximum, minimum, etc.) of all schemes. Considering AUC being the key metric, we summarized the average AUCs grouped by different factors (feature selection strategy, machine learning model, and sampling method). We also conducted a Delong test [59] to evaluate the impact of different methods on predicting results. The variables involved in the study include feature selection methods, machine learning methods, sampling methods, and fivefold cross validation. Hence, the difference in AUC between specific methods can be evaluated by controlling other variables unchanged. *P* < 0.05 is considered statistically significant. In addition, the between-groups sum of squares (BGSS), within-groups sum of squares (WGSS), and total sum of squares (TSS) were used to measure deviation of the AUCs grouped by machine learning models, sampling methods, and feature selection strategies, and their definitions are given as follows:

(1) $$\begin{array}{c} \text{BGSS}=\sum_{i=1}^{r}n_{i}{\left({\bar{x}}_{i}-\bar{x}\right)}^{2},\\ \text{WGSS}=\sum_{i=1}^{r}\sum_{j=1}^{n_{i}}{\left({\bar{x}}_{i}-x_{ij}\right)}^{2},\\ \text{TSS}=\sum_{i=1}^{r}\sum_{j=1}^{n_{i}}{\left(\bar{x}-x_{ij}\right)}^{2}=\text{WGSS}+\text{BGSS,} \end{array}$$

where *r* refers to the number of groups, *n*_*i*_ refers to the number of examples belonging to group *i*, $\bar{x}$ refers to the mean of all samples, ${\bar{x}}_{i}$ refers to the mean of *i*^th^ group, and *x*_*ij*_ refers to the *j*^th^ sample of the *i*^th^ group. Given certain TSS, the larger the GBSS (the less the WGSS), the better the grouping. The experiments implemented were based on R software (version 3.61); the identification was conducted with the “caret” packages.

## 3. Results

We analyzed the experimental results in both scheme and factor level.

### 3.1. Analysis at Scheme Level

The schemes were mainly measured by averaging mentioned metrics of the fivefold cross validation, and the top 15 schemes in the test set are shown in Table 3, in descending order of average AUC. A model is considered as considerable predictive performance, if it is of a higher than 0.7 AUC [60, 61]. All NRIs were measured compared to the scheme of RF, backward selection strategy, and original sampling. Table 3 indicates the following: (1) The RF model with original sampling using backward selection strategy achieved the best performance according to accuracy (0.8578) and AUC (0.7199). (2) All top 9 schemes were of RF models, and RF model accounted for 11 of the top 15. Meanwhile, the schemes with a higher than 0.7 AUC were all RF models. (3) For the sampling method, original sampling and oversampling both accounted for 6 in the top 15 schemes, and the top 4 were original sampling. For the schemes with a higher than 0.7 AUC, both oversampling and original sampling accounted for half of all (4) For the NRI, there were 12 schemes with negative results, indicating that their performance was worse than the first one. Only two schemes achieved the positive NRI results, but differences were quite small (RF, original strategy, and original sampling: 0.0020; RF, importance-based strategy, and original sampling: 0.0057).

In addition, the statistics of each metric over the 75 schemes are shown in Table 4. According to Table 4, we can find the following: (1) for all the schemes, the specificity and NPV were quite high, with an average value of more than 0.75 (specificity: 0.8751, NPV: 0.7760), and the maximum value of NPV was 0.9988. In comparison, the sensitivity and PPV values were relatively small, whose mean values are less than 0.4 (sensitivity: 0.3215, PPV: 0.3938). (2) For each scheme, the standard deviations of AUC and specificity were small (AUC: 0.0430; specificity: 0.0208), which means that the values of them are stable.

### 3.2. Analysis at Factor Level

AUC is a useful metric that comprehensively reflects the performance of the model. The average AUCs grouped by each factor (feature selection strategy, machine learning model, and sampling method) are shown in Table 5. The average AUCs grouped by feature selection strategy indicate the following: (1) schemes using LASSO-based strategy had the largest AUC mean (mean: 0.6582), and these using forward selection strategy had the smallest (mean: 0.6426). However, the difference is quite small (0.0156). (2) In terms of standard deviations, except for the forward selection strategy (standard deviation: 0.0626), other strategies are of little difference between each other, and all of them were less than 0.0450. (3) The range (gap between maximum and minimum) of average AUC value of each strategy was around 0.2220.

The average AUCs grouped by machine learning model indicate the following: (1) RF model had the largest AUC mean (mean: 0.6889). (2) The ascending standard deviations were 0.0222 (LR), 0.0256 (XGBoost-tree), 0.0259 (NNET), 0.0314 (RF), and 0.0668 (SVM-linear models). (3) Compared with the other models, the average AUC of the RF model had the largest maximum (max: 0.7355).

The average AUCs grouped by sampling method indicate the following: (1) for oversampling and original sampling methods, AUC had the largest and the least mean values, respectively (oversampling: 0.6604; original sampling: 0.6460). (2) Among the three sampling methods, undersampling achieved the least standard deviation (standard deviation: 0.0354).

For comprehensively evaluating the performance of the factors mentioned above, one-sided Delong tests were conducted on the ROCs of each paired performance group; and the superiority index, which refers to the percentage of results of a certain group which precedes that of another group, is used to indicate the superiority between each factor. The superiority indexes are summarized in Tables 6–8 in the aspect of feature selection strategy, machine learning models, and sampling method, respectively, and only the factor-comparison groups with more than 1/2 superiority index were analyzed accordingly.

According to Tables 6 and 8, feature selection methods and sampling methods show no factor-comparison group with a more than 1/2 superiority index, which indicates that there is no factor (such as oversampling) superior to another factor (such as undersampling) with a threshold of 1/2.  Table 7 presents the superiority index on machine learning models, and it indicates the following: (1) Compared with other machine learning methods, the superiority indexes of RF compared with other machine learning methods are all more than 1/2 (RF versus XGBoost-tree: 45/75, RF versus SVM-linear-tree: 56/75, and RF versus NNET: 49/75), except for the LR; however, the superiority index of RF compared to LR is 35/75, which is very close to 1/2 and much higher than that of LR compared to RF. The analysis above indicates the superiority of RF. (2) All superiority indexes of other machine learning methods compared to SVM-linear are more than 1/2, which indicates the inferiority of SVM-linear.

Table 9 summarized the BGSS, WGSS, and TSS of AUCs grouped by three different factors mentioned above and indicated the following: (1) The maximum of BGSS (0.3191) and minimum of WGSS (0.5376) were obtained by machine learning models' grouping, which accounted for 37.25% and 62.75% of TSS, respectively. (2) The BGSS and WGSS grouped by sampling method were similar to the counterparts grouped by feature selection strategy (BGSS and WGSS grouped by sampling method: 0.0132 and 0.8435; BGSS and WGSS grouped by feature selection strategy: 0.0123 and 0.8443).

## 4. Discussion

The present results indicate the feasibility and robustness of identifying elective urologic surgeries with high cancellation risk. The average AUCs in the test set exceeded 0.65, with the maximum of AUC (0.7199, RF, original sampling, and backward selection strategy).

It is worth noting that RF model accounted for 11 of the top 15 among the 75 schemes, and the schemes with a higher than 0.7 AUC were all RF models. In addition, RF model was significantly different from the other models in the aspect of AUC. Finally, machine learning model factor achieved the maximum of BGSS and the minimum of WGSS. Hence, the selection of machine learning models is considered a key factor in identification of surgeries with high cancellation risk.

Among the top 8 schemes, the first four and the last four were original sampling and oversampling, respectively. However, sampling methods show no significant difference with each other according to the Delong test. In addition, there were large WGSS and small BGSS when grouped by sampling methods. In summary, sampling method is the factor that affects the identification of surgeries with high cancellation risk, but not as important as the machine learning methods, to some extent.

For different feature selection strategies, differences between their means were little and insignificant. In addition, there were large WGSS and small BGSS when grouped by sampling methods. Hence, feature selection strategy is not an important factor that affects the identification of surgeries with high cancellation risk.

This study has limitations. It only focused on the elective urologic surgeries in one hospital, which means that the data are single-centered. Although our predictors covered five information categories that previous studies have covered and on which good results have been obtained, there are also potentially useful predictors that have not been collected. Further research can consider conducting multicenter studies, including multiple hospitals and departments.

## 5. Conclusion

This study provided effective methods for the identification of surgeries with high cancellation risk based on machine learning models and analyzed the key factors that affect the identification of surgeries with high cancellation risk. It proved the feasibility and robustness of identifying surgeries with high cancellation risk, with the considerable maximum of AUC (0.7199) for RF with original sampling using a backward selection strategy. In addition, two-sided test and sum of square error analysis were conducted to measure the effects of feature selection strategy, machine learning model, and sampling method on the identification of surgeries with high cancellation risk; and the selection of machine learning model was identified as the key factors that affect the identification of surgeries with high cancellation risk. This study offers methodology and insights for identifying the key experimental factors for identifying surgery cancellations, and the insights of it are useful to further research on machine learning-based identification of surgeries with high cancellation risk, in designing experimental process.

## Figures and Tables

**Figure 1:** Experiment flowchart.

**Table 1:** Predictors collected in this study.

Category	Number of predictors	Predictor(s)
Patients' information	4	Name, age, sex, and AT
Admission information	4	NDA, visit number, identification number of patient, and register number
Workup information	7	Drug allergy, names of drugs administered, blood type, WHSB, SN, and ST
Surgery schedule information	7	ONS, OR, surgery date, surgery time, surgeon, NSOD, WSHSB, and purpose of surgery
Administrative issues	10	Operation staff, department, ward, BD, last updated time, staff who last updated the information, WSDLH, WMSD, WC, and surgery expenditure
Surgery process records	23	Actual date/time when surgery began/ended, actual date/time when patient left OR, actual date when anesthesia was started, actual time when anesthesia was ended, actual date/time when predictive medicine was administered, body temperature, blood transfusion in surgery, autologous blood, allogeneic blood, plasma, thrombocyte, pathological examination, state of consciousness, general skin conditions, special skin conditions, drainage situation, surgery item delivery, anesthesia degree, and surgical incision category

AT: anesthesia type. BD: bed number. NDA: number of days admitted. NSOD: number of surgeries in the OR on the day. ONS: order number of surgery. OR: operating room. SN: surgery name. ST: surgery type. WC: whether surgery is cancelled. WHSB: whether there has been a surgery before. WMSD: whether it is the main surgery day. WSDLH: whether the surgery day is a legal holiday. WSHSB: whether the surgeon has surgery before.

**Table 2:** Predictors considered in this study.

Category	Number of predictors	Predictor(s)
Patients' information	3	Age, sex and AT
Admission information	1	NDA
Workup information	2	WHSB and ST
Surgery schedule information	5	OR, surgeon, NSOD, ONS, and WSHSB
Administrative issues	3	WSDLH, WMSD, and WC

AT: anesthesia type. NDA: number of days admitted. NSOD: number of surgeries in the OR on the day. ONS: order number of surgery. OR: operating room. ST: surgery type. WC: whether surgery is cancelled. WHSB: whether there has been a surgery before. WMSD: whether it is the main surgery day. WSDLH: whether the surgery day is a legal holiday. WSHSB: whether the surgeon has surgery before. Predictor(s): predictors mentioned above were preliminarily identified through expert interviews.

**Table 3:** Top 15 schemes in the test set.

	Model	Strategy	Sampling	AUC	Accuracy	Sensitivity	Specificity	PPV	NPV	NRI
1	RF	Backward selection strategy	Original sampling	0.7199	0.8578	0.6712	0.8668	0.1963	0.9819	0.0000
2	RF	Original strategy	Original sampling	0.7136	0.8574	0.6740	0.8660	0.1901	0.9826	0.0020
3	RF	Forward selection strategy	Original sampling	0.7135	0.8560	0.6284	0.8692	0.2173	0.9759	−0.0404
4	RF	Importance-based strategy	Original sampling	0.7131	0.8574	0.6783	0.8654	0.1852	0.9835	0.0057
5	RF	Backward selection strategy	Oversampling	0.7055	0.8343	0.4579	0.8722	0.2654	0.9411	−0.2079
6	RF	Forward selection strategy	Oversampling	0.7034	0.8154	0.3904	0.8736	0.2963	0.9129	−0.2740
7	RF	Importance-based strategy	Oversampling	0.7029	0.8398	0.4869	0.8720	0.2580	0.9490	−0.1791
8	RF	Original strategy	Oversampling	0.7018	0.8394	0.4874	0.8726	0.2630	0.9476	−0.1780
9	RF	Forward selection strategy	Undersampling	0.6847	0.6176	0.2369	0.9003	0.6383	0.6137	−0.4008
10	NNET	LASSO-based strategy	Original sampling	0.6814	0.8398	0.4167	0.8424	0.0123	0.9934	−0.2789
11	RF	Backward selection strategy	Undersampling	0.6814	0.6328	0.2436	0.9009	0.6284	0.6336	−0.3935
12	RF	Original strategy	Undersampling	0.6808	0.6310	0.2384	0.8960	0.6074	0.6355	−0.4036
13	SVM-linear	LASSO-based strategy	Oversampling	0.6797	0.6597	0.2523	0.8970	0.5877	0.6732	−0.3887
14	LR	LASSO-based strategy	Oversampling	0.6794	0.6457	0.2493	0.9012	0.6185	0.6508	−0.3875
15	LR	LASSO-based strategy	Original sampling	0.6793	0.8429	0.5492	0.8459	0.0346	0.9947	−0.1429

LR: logistic regression model. NNET: neural networks. RF: random forest. SVM-linear: support vector machine-linear. XGBoost-tree: extreme gradient boosting-tree. Accuracy: ratio of the correctly predicted sample number to the total predicted sample number. Sensitivity: ratio of correctly predicted positive samples to the total number of true positive samples. Specificity: ratio of correctly predicted negative sample number to the total number of true negative samples. PPV: positive predictive value. NPV: negative predictive value. AUC: area under the receiver operating characteristic curve. NRI: net reclassification index; all NRIs were measured compared to the scheme of RF, backward selection strategy, and original sampling. The values in the table are averages of the fivefold cross validation.

**Table 4:** Statistics on the performance metrics.

	Max	Min	Mean	St. Dev.
AUC	0.7199	0.5310	0.6537	0.0430
Accuracy	0.8578	0.5967	0.7166	0.1016
Sensitivity	0.6783	0.1736	0.3215	0.1360
Specificity	0.9012	0.8419	0.8751	0.0208
PPV	0.6383	0.0031	0.3938	0.2362
NPV	0.9988	0.5914	0.7760	0.1634

Accuracy: ratio of the correctly predicted sample number to the total predicted sample number. Sensitivity: ratio of correctly predicted positive samples to the total number of true positive samples. Specificity: ratio of correctly predicted negative sample number to the total number of true negative samples. PPV: positive predictive value. NPV: negative predictive value. AUC: area under the receiver operating characteristic curve.

**Table 5:** Statistics on AUCs grouped by different factors.

Grouping factors	Groups	*N*	Mean	St. Dev.	Min	Pctl(25)	Pctl(75)	Max	Range
*Feature selection strategy*	Original strategy	75	0.6547	0.0428	0.5125	0.6372	0.6819	0.7292	0.2167
	LASSO-based strategy	75	0.6582	0.0441	0.4948	0.6449	0.6821	0.7239	0.2291
	Forward selection strategy	75	0.6426	0.0626	0.5085	0.6307	0.6846	0.7355	0.2270
	Backward selection strategy	75	0.6580	0.0427	0.5152	0.6435	0.6788	0.7331	0.2179
	Importance-based strategy	75	0.6550	0.0436	0.5125	0.6350	0.6823	0.7307	0.2182

*Machine learning model*	RF	75	0.6889	0.0314	0.6100	0.6713	0.7129	0.7355	0.1255
	LR	75	0.6666	0.0222	0.6297	0.6514	0.6792	0.7161	0.0864
	XGBoost-tree	75	0.6574	0.0256	0.6110	0.6353	0.6748	0.7171	0.1061
	NNET	75	0.6552	0.0259	0.6163	0.6362	0.6702	0.7239	0.1076
	SVM-linear	75	0.6005	0.0668	0.4948	0.5360	0.6558	0.7184	0.2236

*Sampling method*	Oversampling	125	0.6604	0.0403	0.5085	0.6385	0.6908	0.7355	0.2270
	Undersampling	125	0.6548	0.0354	0.5085	0.6398	0.6756	0.7239	0.2154
	Original sampling	125	0.6460	0.0626	0.4948	0.6365	0.6911	0.7340	0.2392

*N*: number of cases. Mean: mean value corresponding to AUC of each model. St. Dev.: standard deviation corresponding to AUC of each model. Pctl(25): AUC corresponds to the first quartile of the variance numerical distribution of each model. Pctl(75): AUC corresponds to the third quartile of the variance numerical distribution of each model. LR: logistic regression model. NNET: neural networks. RF: random forest. SVM-linear: support vector machine-linear. XGBoost-tree: extreme gradient boosting-tree.

**Table 6:** Superiority index of Delong test on AUCs grouped by feature selection strategies.

	Original strategy	LASSO-based strategy	Forward selection strategy	Backward selection strategy	Importance-based strategy
Original strategy	NA	23/75	8/75	8/75	24/75
LASSO-based strategy	13/75	NA	10/75	11/75	14/75
Forward selection strategy	11/75	21/75	NA	13/75	11/75
Backward selection strategy	0/75	18/75	5/75	NA	10/75
Importance-based strategy	11/75	21/75	2/75	10/75	NA

NA: not available.

**Table 7:** Superiority index of Delong test on AUCs grouped by machine learning model.

	RF	LR	XGBoost-tree	SVM-linear	NNET
RF	NA	7/75	4/75	3/75	5/75
LR	35/75	NA	2/75	0/75	1/75
XGBoost-tree	45/75	7/75	NA	1/75	2/75
SVM-linear	56/75	48/75	46/75	NA	46/75
NNET	49/75	12/75	5/75	7/75	NA

LR: logistic regression model. NNET: neural networks. RF: random forest. SVM-linear: support vector machine-linear. XGBoost-tree: extreme gradient boosting-tree. NA: not available.

**Table 8:** Superiority index of Delong test on AUCs grouped by sampling method.

	Oversampling	Undersampling	Original sampling
Oversampling	NA	8/125	18/125
Undersampling	18/125	NA	25/125
Original sampling	20/125	18/125	NA

NA: not available.

**Table 9:** Analysis of sum of square error.

	TSS	BGSS	BGSS/TSS (%)	WGSS	WGSS/TSS (%)
Grouped by feature selection strategy	0.8567	0.0123	1.44	0.8443	98.55
Grouped by ML model	0.8567	0.3191	37.25	0.5376	62.75
Grouped by sampling method	0.8567	0.0132	1.54	0.8435	98.46

TTS: total sum of square error. BGSS: between-groups sum of square error. WGSS: within-groups sum of square error.

## Data Availability

The data supporting the study findings will not be shared since it is an organizational property. Data were anonymous, and study subjects could not be identified.
